This article has been retracted.

# Evaluation and Analysis of Traditional Customary Law Based on the Perspective of Big Data

**DOI:** 10.1155/2022/5088630

**Published:** 2022-06-14

**Authors:** Juanjuan Yang, Tee Boon Chuan

**Affiliations:** ^1^Institute of Chinese Studies, Universiti Tunku Abdul Rahman, 43000 Kajang, Malaysia; ^2^School of Marxism, HaiKou University of Economics, Haikou, 571000 Hainan, China

## Abstract

Today's rule of law construction in China is walking between the conflict and coordination of factors such as reality and ideals, tradition and modernity, local and foreign, and local knowledge and universal principles, all while continuing to strengthen the unification of the legal system and advance the modernization of the rule of law. Traditional customary law, which is the most representative local resource culture, is unquestionably one of the most important themes in the formation of the rule of law. It has far-reaching significance for the development of ethnic jurisprudence, the reunderstanding of traditional culture, and the construction of ethnic unity and harmonious society. Based on this background, this paper uses big data technology to collect relevant experimental data and proposes a traditional customary law value assessment based on BPNN. The completed work is as follows: (1) this paper clarifies the concept of customary law and the difference between it and related concepts and introduces the domestic relevant research on traditional customary law and the interactive relationship between customary law and national law in dynamic legal practice and puts forward the status and influence of customary law in contemporary legal practice. (2) The related technologies of neural network are introduced, and a traditional customary value evaluation system that can be used for experiments is constructed. (3) Experiment with the designed data set to see if the BP model is feasible. The experimental results suggest that the model proposed in this study has a low error rate and performs well while evaluating traditional common law values.

## 1. Introduction

My country's legal circles have paid attention to customary law mainly since the 1990s. The study of Chinese customary law is mainly influenced by the western postmodern thought, which has formed the postmodern legal theory in the field of law. The core idea of postmodern legal theory holds that rational individuals as autonomous legal subjects do not exist, and modern society is illusory. People in the present social system are not “actual people,” but appendages of the social structure, and the manner of their existence is rights [1, 2]. The universality of the law is a virtual “macrodiscourse,” and the principles in the law are only an assumption. The process of modernizing the rule of law is also a process of training people to abandon specific and individual experiences, accept general rules, abandon the rich and colorful human life, and accept standardized behavior patterns. Modern law has been influenced by postmodern jurisprudence. Individuals are independent, conscious, rational subjects, according to modern law [3]. Law progresses from lower to higher levels, and truth can be discovered by trial and error. Postmodern legal theory has brought methodological innovation to the legal circle in our nation which was previously dominated by modern legal theory and has extended the boundaries of legal research. The study of traditional customary law has caused a lot of disputes in the academic circles. Scholars hold different views on issues ranging from whether customary law is law to what is the significance of customary law to the construction of the rule of law. Domestic legal history and legal sociology scholars are the main force in the study of traditional customary law, and their research methods are mainly to find answers from historical materials or start with the grass-roots judicial system, analyze the influence of customary law on grass-roots judicial adjudication, and study the interaction between traditional customary law and statutory law [4]. There are also scholars who doubt the practical significance of customary law research and even believe that customary law research is not only meaningless to the construction of the rule of law, but will even hinder the process of the construction of the rule of law. In view of the fact that a truly independent space for academic research has not yet been formed, it is generally believed that academic research should have practical significance, so this criticism also has considerable deterrence. Therefore, this article intends to give a little answer to this criticism. Although I do not agree that academic research must have so-called practical significance, I must insist on showing the truth of the facts. The issue of traditional customary law has such great significance to contemporary legal practice, and even the neglect of this issue is the crux of the repeated obstruction of the rule of law process [5]. Criticisms about traditional customary law research are inseparably linked to the current state of traditional customary law research. The current research is mainly carried out from a historical perspective, and some scholars describe the situation of customary law in rural justice from an empirical perspective, but they all give people a negative impression [6]. Traditional customary law is a phenomenon that has existed in history or still exists in areas where the rule of law is underdeveloped. Such research results inevitably lead to the view that traditional customary law is backward and contradicts the modernization of the rule of law, which is actually a misunderstanding of traditional customary law [7, 8]. Based on the shortcomings and misunderstandings of the current traditional customary law research, the main content of this paper is to discuss the important role of traditional customary law in legal practice, especially to reveal the operation of customary law in a modern rule of law society or developed areas under the rule of law. The reason forces us to reconsider the meaning and direction of the rule of law's modernization. Because theoretical circles have yet to form a unified authoritative view on the basic theory of customary law, this paper begins with the fundamental concept of traditional customary law, defines the concept and main characteristics of customary law, and distinguishes customary law from related concepts. In modern legal practice, the interaction between customary and national law is primarily expressed in the relationship between the two. Traditional customary law and national law are transformed into each other in legal practice. This interactive relationship may have a certain impact on the construction of the rule of law. In this context, based on big data technology, this paper uses neural network technology to evaluate and analyze the value of traditional customary law, so as to reveal the significance of traditional customary law to the construction of the rule of law in my country.

The following is the paper's organization paragraph: Section 2 discusses the associated work. The techniques of the proposed notions are examined in Section 3. The trials and results are discussed in Section 4. Finally, the research job is completed in Section 5.

## 2. Related Work

In a sense, the history and achievements of foreign legal circles studying customary law are mainly reflected in the field of legal anthropology. Therefore, it is necessary to review and sort out the history and development of legal anthropology in detail. Legal anthropology is a discipline at the edge of the two major disciplines of law and anthropology. It is a new discipline that jurists and anthropologists “interpenetrate” and cultivate on the edge of their respective disciplines [9]. For a jurist, the main sources of many legal formulations, revisions, and procedures, and their universal application, are found in the concepts and relationships embodied in everyday social life. It is this kinship between law and anthropology that drives anthropologists' attention to law. It also promotes jurists to attach importance to anthropological materials and methods and gradually forms an “emerging” interdisciplinary subject [10]. Reference [11] presents what he calls “relative, contingent relationships” that affect the legal basis, including climatic conditions, geographic environment, religious beliefs, and the political structure of a particular country. If the laws of one country can be adapted to another country, it is only very coincidental. Reference [12] believes that law is deeply rooted in the history of a particular nation, depends on the national spirit and national consciousness, and regards law as a part of the whole of social existence. From the perspective of discussing the status and role of the early human legal system in individuals of different civilizations, the dynamic research provides theoretical support. Reference [13] conducted field research and published “Crime and Customs in Primitive Society” in 1926, which is of epoch-making significance for the development of legal anthropology and the study of traditional customary law. Reference [14] believes that there is customary law, and divides the law into three types: customary law, bureaucratic law, and legal order. Reference [15] presents a very different view. In a broad sense, customary law secretly makes new laws, like the latent life of plants and animals before they are born, it is the life force of legal rules, its scope of application is infinite, and it is no exaggeration to say that it is the only source of law. Reference [16] identifies customary law as one of the two basic types of law alongside statute law and argues that customary law arises from an act generally observed where the actor does not consciously aim to create the law, but they must see their actions as conforming to binding norms rather than arbitrary choices, and customary law is equally valid. Reference [17] analyzes the meaning of custom for the formation of law, and the transitional boundaries between custom and custom and law. Reference [18] conducted a comparative analysis of the external order and the internal order and conducted a comprehensive study of customary law including customs and conventions when discussing the internal order. For a long time, due to the constraints of the class view and the influence of the monistic theory of law, when discussing the creation of law and the origin of law, the legal circle in my country always believed that customary law was associated with the state, unique to class society, and recognized by the state. And the habit of implementation is guaranteed by the coercive force of the state, while ignoring the objective existence of customary law and denying the category of customary law as law [19]. In the middle and late twentieth century, with the accelerated pace of reform and opening up, my country's humanities, social sciences, and other exchanges with the international community have increased, and the academic atmosphere has been unprecedentedly active. Domestic scholars began to reexamine the legal theory and research methods in our country, and more and more jurists advocated that the study of law should be related to a specific society, culture, system, etc. The de facto existence of customary law and legal pluralism has become an indisputable issue. Scholars have begun to focus on the analysis of the cultural background, functional mode, generation, and operation mechanism of customary law, especially the fate of customary law in the trend of legal unification, which is a hot spot that people are highly concerned about. Reference [20] expands the research horizon to the customary law of ethnic clans and villages, the customary law of industry, the customary law of religious monasteries, and the customary law of secret societies. It points out that minority customary law still largely dominates the minds of local people and is an effective mode of social control in minority areas. Reference [21–23] upholds the concept of legal pluralism and uses the concept of “folk law” from the perspectives of social, historical, and legal anthropology and combines a large number of rich historical facts and community cases. It makes an in-depth analysis of the status and function, operation and practice, and development and trend of national law and traditional customary law in rural society. Obviously, the views of the above parties cannot be reached, and the research methods used are also different, but most scholars recognize the existence of customary law and accept the fact of “law pluralism.” The research at this stage simply points out the relationship between traditional customary laws as a supplement to national law, but has never found a satisfactory solution to the problem of where customary law goes, thus revealing the significance of traditional customary law to the construction of the rule of law in our country.

## 3. Method

In this chapter, we discuss the introduction to artificial neural networks, network structure of BP neural network, the algorithm principle of BP neural network, deficiencies and improvements of BP neural network algorithm, and traditional and customary law value assessment system in depth.

### 3.1. Introduction to Artificial Neural Networks

The field of brain research developed the ANN data processing paradigm after studying biological neural networks in the brain. The human brain is a biological network structure made up of billions of neurons connected by complicated interconnections, as we all know. It is the source of tools for humans to carry out a series of daily activities such as memory, analysis, reasoning, and recognition. The processing speed of data information is also much higher than the processing speed of today's fastest computers. The basic unit of work of neural network in biology is biological neuron composed of cell body and synapse. The intensity also changes continuously with the change of external stimuli, thereby realizing information storage and memory. When we see a familiar face or hear a familiar voice, it only takes a few hundred milliseconds for the biological neural network system to recognise it, which is a series of events. This ability of biological nerves, however, is not innate. Our brains have been constantly receiving information from the external environment since birth, and the connections between neurons in the brain are constantly altering, allowing us to store a great quantity of data. It is a learning process, and ultimately realize various mental activities such as thinking and emotions through these. Analogous to the behavior of information storage and processing of neurons in the human brain, an ANN model composed of a large number of artificial neurons through a certain connection method can theoretically achieve functions similar to biological neural networks. Neurons change their own structure by continuously receiving the “stimulation” of external data information, that is, the connection mode and connection strength between neurons. This change is reflected in the ANN as a change in the connection weight between neurons, through this change to process the input data information to achieve “learning” behavior. The ANN is realized by linear weighting and function mapping of the input signal, and the weight adjustment process is realized by a suitable learning algorithm to replicate the process of biological nerve cells receiving stimulation from other cells and creating output nerve signals. The data processing model established in this way is the ANN model. Although this bionic mathematical model is far from the true biological neural network, the current research results have been successfully applied to many solutions to practical problems.

### 3.2. Introduction to BP Neural Network

The neural network model can be divided into two types of network structure: feed-forward and feedback. In the feed-forward network structure, the neuron nodes of each layer will receive the input data of the previous layer and then use the linear weighting method to output the output as the input of the next layer through the function mapping. The whole process data flows in only one direction. Without the step of data feedback, the BPNN belongs to the feed-forward neural network. According to the learning method, the neural network model can be divided into supervised learning and unsupervised learning. Supervised learning means that the training and learning of the model need to be guided by the determined output data, so that the model can learn the relationship between the input and output values. The unsupervised model does not need it, and the algorithm of the BPNN belongs to the former. The BPNN is the core and essence of the entire ANN and has shown good performance in various fields such as identification, regression, and classification. Therefore, about 80% of the neural network models in practical applications take the form of BPNN or its related.

#### 3.2.1. Network Structure of BP Neural Network

As a feed-forward neural network model, BPNN model consists of three parts: input layer, hidden layer, and output layer. The hidden layer can have one or more layers, unlike the input and output layers, which both have just one layer. This article uses a single hidden layer to demonstrate the basic structure of the BPNN model, as shown in Figure 1, where *x*_*A*_ is the network structure's input data. *I* is the input layer of the network structure, *W*_*ab*_ is the connection weight of the input layer parameters to the hidden layer node, *H* is the hidden layer of the network structure, *W*_*bc*_ is the connection weight of the hidden layer node to the output layer node, *O* is the output layer of the network structure, and *y*_*c*_ is the actual output of the network structure.

#### 3.2.2. Characteristics of BP Neural Network

In order to analyze the relationship between the input and the output in the BPNN, the network output is obtained by inputting the input data into the network model through the forward algorithm, and the error function between the actual output and the expected output of the network is established, also called the loss function. The function approximation can be achieved by continuously optimizing the algorithm to obtain the minimum value of the loss function, thereby reflecting the relationship between the input and output parameters. The specific algorithm principle and weight adjustment process will be given in the next section. The characteristics of the BPNN model can be roughly summarized as the following three points:

1. The network structure is composed of multiple layers, and there is no connection between all the neuron nodes in the same layer, and each adjacent layer has the connection which is fully connected, that is, all neuron nodes in the previous layer are connected to all neuron nodes in the next layer. This multilevel structure design can mine a large amount of information from the input data to complete complex tasks
2. The BPNN adopts the error back propagation algorithm. The input data is input from the input layer and propagates forward layer by layer through the hidden layer to the output layer. After reaching the output layer, an error function is established, and the error reaches the input layer through the hidden layer, and the backward propagation in the reverse direction layer by layer continuously corrects the connection weights of the network. By iterating this process many times, you can eventually make the error smaller and smaller
3. Since the BPNN model needs to use the gradient descent algorithm to optimize the model, it is necessary to solve the partial derivative of the loss function. When no activation function is set, the neural network model is actually a linear weighting of parameters. When a differentiable activation function is set, the gradient descent algorithm can be used to optimize the model

### 3.3. The Algorithm Principle of BP Neural Network

As shown in Figure 2, we assume that there are an input neural parameters *x*_1_, *x*_2_, *x*_3_, ⋯*x*_*A*_, which are represented as [*x*_1_, *x*_*A*_] in the form of a matrix, and the input information and output information of each layer are represented by *M* and *N*, respectively, then the input information of the input layer is also the input information of the entire network, which can be expressed as:

(1) $$\begin{array}{c} M_{I}=\left[x_{1},x_{A}\right]. \end{array}$$

The output information of the input layer is:

(2) $$\begin{array}{c} N_{I}=M_{I}=\left[x_{1},x_{A}\right]. \end{array}$$

Assuming that there are *B* neuron nodes in the hidden layer, the input of the *b*th neuron node of the hidden layer can be expressed as the weighted sum of the output *N*_*I*_ of the input layer and the sum of the bias term parameter *p*:

(3) $$\begin{array}{c} M_{H}^{b}=\overset{A}{\underset{a=1}{\sum }}W_{ab}∙N_{I}^{a}. \end{array}$$

Assuming that the activation function of the hidden layer is *f*, then the output of the *b*th neuron node of the hidden layer can be expressed as:

(4) $$\begin{array}{c} N_{H}^{b}=f\left(M_{H}^{d}\right). \end{array}$$

Assuming that there are *C* neuron nodes in the output layer, the input of the *c*^th^ neuron node of the output layer can be expressed as the weighted sum of the output of the hidden layer and the sum of the bias term parameters:

(5) $$\begin{array}{c} P_{O}^{c}=\overset{B}{\underset{b=1}{\sum }}W_{bc}∙N_{H}^{b}+k. \end{array}$$

Assuming that the activation function of the output layer is *g*, then the output of the *c*^th^ neuron node of the output layer, that is, the output of the network structure can be expressed as:

(6) $$\begin{array}{c} y_{c}=N_{O}^{c}=g\left(P_{O}^{c}\right). \end{array}$$

In this way, we put input neural parameters *x*_1_, *x*_2_, *x*_3_, ⋯*x*_*A*_ into the network structure, and the output of the network is *y*_1_, *y*_2_, *y*_3_, ⋯*y*_*c*_. Assuming that the expected output of the network structure is *P*_1_, *P*_2_, *P*_3_, ⋯*P*_*C*_, and the error of the cth neuron node of the output layer is *E*_*c*_. It can be expressed as:

(7) $$\begin{array}{c} E_{c}=P_{c}-y_{c}. \end{array}$$

The total error *E* of the network is the loss function, which can be expressed by the mean square error formula as:

(8) $$\begin{array}{c} E=\frac{1}{C}\overset{C}{\underset{c=1}{\sum }}E_{c}^{2}. \end{array}$$

After the loss function of the network is obtained, the correction of the weights corresponding to the network parameters needs to be determined according to the loss function. The gradient of the loss function to the weight is calculated by the steepest descent method, and the weight is adjusted in the opposite direction of the gradient. The whole process is divided into two steps:

1. Adjust the connection weight *W*_*bc*_ from the hidden layer node to the output layer node
2. Adjust the connection weight *W*_*ab*_ from the input layer node to the hidden layer node. Make adjustments to *W*_*bc*_. First, the formula for calculating the adjustment of the loss function to the weights is:

(9) $$\begin{array}{c} ∆W_{bc}=-\mu \frac{\partial E}{\partial W_{bc}}, \end{array}$$

where *μ* is the step size of each adjustment of the weight, also called the learning rate.

Then, the expression of the relationship between the adjusted weight *W*_*bc*_(*n* + 1) and the adjusted weight *W*_*bc*_(*n*) is:

(10) $$\begin{array}{c} W_{bc}\left(n+1\right)=W_{bc}\left(n\right)+∆W_{bc}. \end{array}$$

In the process of adjusting the connection weight *W*_*bc*_ from the hidden layer node to the output layer node, *N*_*H*_^*b*^ is the output value of the hidden layer node neuron, which can be regarded as an independent variable, and defines the concept of local gradient *λ*_*O*_^*c*^, which represents the required change in weights. The expression for the local gradient is:

(11) $$\begin{array}{c} \lambda_{O}^{c}=\frac{\partial E}{\partial M_{O}^{c}}=\frac{\partial E}{\partial E_{c}}∙\frac{\partial E_{c}}{\partial y_{c}}∙\frac{\partial y_{c}}{\partial M_{O}^{c}}=-2E_{c}g^{\prime }\left(M_{O}^{c}\right). \end{array}$$

Then, the amount of each adjustment of the weights can be expressed as:

(12) $$\begin{array}{c} ∆W_{bc}=2\mu \lambda_{O}^{c}N_{H}^{b}. \end{array}$$

Adjust the connection weights *W*_*ab*_ of the connection weights from the input layer nodes to the hidden layer nodes. Similar situation with *W*_*bc*_

(13) $$\begin{array}{c} ∆W_{ab}=2\mu \lambda_{H}^{b}N_{I}^{a}. \end{array}$$

In this way, the connection weights from the hidden layer nodes to the output layer nodes and the connection weights from the input layer nodes to the hidden layer nodes are adjusted in one round, and the error back propagation process of the first round is completed. The more complicated step in the whole process is that when adjusting the weight between the input layer and the hidden layer, since the hidden layer is invisible, the calculation of the local gradient needs to use the local gradient calculated in the previous step, that is, between the hidden layer and the output layer. The local gradient of BPNN can only be reversed in the process of weight adjustment. After adjusting and updating the weights of the network, a new error function is obtained through the forward propagation of the input information for the next round of weight adjustment. Through repeated iterations, the network error can be continuously reduced and the input is continuously approached. The functional relationship with the output, so as to realize the network function to achieve the purpose of classification or prediction.

### 3.4. Deficiencies and Improvements of BP Neural Network Algorithm

#### 3.4.1. Disadvantages of BP Algorithm

Although the BP algorithm can approximate any complex functional relationship with arbitrary precision in theory, with more and more use, some shortcomings are gradually discovered, which are roughly summarized as more parameters, easy to fall into the local optimal solution and the three points of overfitting phenomenon:

1. The problem of more parameters. BPNN needs more parameters due to its structural characteristics, and the determination methods of many parameters are not very certain. Layer weights and learning rates, as well as the number of nodes in each nested layer, are all included in this list. When utilizing the BP method, the phenomena of “gradient diffusion” may arise if the number of network levels is too deep. Overlearning will occur if the number of nodes in the hidden layer is excessive. There is a risk of poor learning if the number of neurons is too low. As a result, if the learning rate is too high, the parameters may swing back and forth on either side of the optimum solution but fail to converge, or the learning rate is too little. The optimal solution cannot be quickly converged within the number of iterations
2. The phenomenon of local optimal solution. Due to the setting of the initial weight, the BP algorithm may have a poor “initial position” of the loss function, and the learning process only converges to the local minimum value and does not reach the global minimum value; thus, the phenomenon of local optimal solution appears
3. Overfitting phenomenon. After the BP algorithm optimizes the set loss function on a certain training data set, the model may perform well on the training data, but perform poorly on the unknown data. The reason for this is that the model overly “remembers” each “random noise” part of the training data and neglects to “learn” general trends in the training data

#### 3.4.2. Improved Method of BP Algorithm

Although the BP algorithm has flaws, scientists have continued to explore and improve it, and some enhanced approaches have demonstrated promising outcomes in practice.

1. Regarding the setting of the learning rate, the exponential decay method can be used to set the dynamic learning step size, and a larger learning rate can be set in the early stage of iterative learning to quickly obtain a relatively optimal solution and gradually decrease with the increase of the number of iterations. A small learning rate is used to ensure stable convergence in the end
2. In the case of local optimal solutions, the genetic algorithm can be used to “preprocess” the initial weights instead of using random weights to set the initial parameters, resulting in a loss function “initial position” that is a relatively ideal value, greatly improving the model's stability and better predicting the function's output
3. Regarding the overfitting problem, a regularization method can be used, and indicators can be added to describe the complexity of the model, through the idea of limiting the size of the weights to control that the model cannot arbitrarily learn “random noise” in the training data

### 3.5. Traditional and Customary Law Value Assessment System

In order to establish a reasonable traditional customary law value evaluation system, we must first discuss the value of traditional customary law.

#### 3.5.1. Control of Rural Society

Rousseau has commented on the customary law, adding to these three a fourth, and the most important of all, which is neither inscribed in marble, it is not engraved on the bronze watch, in the folks' hearts. If you want to discover what constitutes a nation's genuine constitution and how the nation's founding spirit may be preserved and replaced, you need to go no further than the power of habit. This is the power of habit. It can be said that customs and customary laws formed based on customs and habits are an important part of ancient Chinese rituals. These customary laws arise from people's daily life and are the norm in people's daily life. Ancient China has a deep understanding of the role of rituals. It can be said that it is the first line of defense to prevent disputes and achieve a good social order, and it is the most important means of social control. From the point of view of the code of conduct alone, this is no different from the law, and the law is also a code of conduct. The difference between ritual and law is the power to maintain norms. The law is enforced by the power of the state. The state refers to political power. Tribes were also political power before the modern state was founded. This tangible authority is not required to keep the ritual going. It is tradition that maintains this norm. In fact, the content of traditional customary law is very rich, and its manifestations are also varied. The basis for its effectiveness may come from tradition and its social organization, or from the state. The source of law is customary law, which is a social norm, and there have been countries in history where a set of carefully formulated customary laws was more than enough to solve problems. Most of the countries in ancient times were rural societies with traditional customary law, so customary law played a central and leading role in their social control system.

#### 3.5.2. Demonstrate Psychological Conviction

Like legal concepts, traditional customary law has many interpretations. In traditional Chinese jurisprudence, all laws are related to the state, and customary law is no exception. Therefore, customary law is a habit recognized by the state and guaranteed by the state's coercive force. It strictly distinguishes custom from customary law, and its scope is narrow. Whether this usage of customary law is appropriate or not is irrelevant. According to general terminology, as a norm of customary law, its effectiveness depends to a large extent on a similar mechanism of enforcement, albeit from consent rather than enactment. Habits are not characterized by any coercive mechanism. The Oxford Dictionary of Law is more open, when some custom and custom and prevailing practice has been established in a considerable part of the country, recognized and regarded as legally binding, as if it were based on written legislative rules, they can rightfully be called customary law. Here, its validity is based on people's “psychological conviction,” as long as people are convinced of its legal effect, it is customary law. This conviction may come from coercive institutions, from natural laws, or from religion, etc.

#### 3.5.3. Improve the Binding Force of Custom

In recent years, Chinese academics have steadily expanded the concept of customary law and collaborated in the research of customary law. In the opinion of some legal academics, national customary law is a code of behavior formed by people based on facts, experience, and a specific social authority that is apart from state statute law. He also summed up the characteristics of national customary law into six characteristics: rooted locality, content vitality, informality of procedure, regionality of jurisdiction, internal control of operation, and constancy of maintenance. Some scholars define customary law as some custom practice and common practice recognized and regarded as legally binding. The sum of customary binding forces that preserve and regulate the relationship between a social organisation and its members is referred to as customary law. It is created by the members of the organisation or group to meet the organizations or group's production and survival demands. Certain regions are subject to mandated codes of behavior. The characteristics and manifestations of customary law are fully explored in “China Minority Customary Law Research,” which has a stronger guiding role in understanding and interpreting customary law. Customary law is corresponding to the statutory law of the state. It comes from various social organizations and social authorities, regulates the behavior of all members of a certain social organization and social area, and is generally abided by them. Secondly, it must be clear that customary law is not created out of thin air; it comes from various habits that already exist in society. Lastly, customary law is both natural and customary, and it is also agreed upon by members of a specific social organization. It can be unwritten or written, and it must not be considered that customary law must be expressed in unwritten form. Customary law mainly relies on word of mouth and behavior to spread and inherit. In addition, some scholars believe that customary law is a code of conduct that is jointly confirmed by members of society and is applicable to a certain area in order to maintain social order, adjust, and deal with people's mutual relations within or between ethnic groups. This article still follows the habit of most Chinese and foreign scholars to call it “customary law” and believes that customary law is a habit of people and their communities in their mutual exchanges, with certain rights and obligations as the content and is established by people outside the country. A code of conduct that guarantees that it is generally followed in a certain area or group.

In this regard, our considerations are: first, the emergence of customary law is based on the premise of people's interaction with each other and is a code of conduct to clarify their mutual rights and obligations, rather than the premise of the formation of a state or other public authority, trying to expand the time limit of its existence as much as possible; second, the inclusion of rights and obligations is to distinguish them from purely obligatory taboos, morals, and other norms, and their rights and obligations are not necessarily very clear and not necessarily equal, so the use of the word “must” is limited; thirdly, the way of enforcement outside the state is to distinguish between customary law and national law; the case law in the common law system and the custom recognized by the national legislative process are not in the scope of customary law, those who do not use “coercive force” but use coercive methods, including unorganized coercive methods such as pressure from religion, spirituality, and social public opinion; fourth, a specific region or community emphasizes that customary law is a type of local knowledge distinct from human beings' universal natural law. For example, it is not a customary law for a group to wear clothes, and it may be a customary law not to wear it, to wear it less, or to wear it uniquely and nonnormative behavior towards specific people and things. To sum up, this paper constructs a traditional customary law value evaluation system, as shown in Table 1. According to the input indicator data, the output is finally set to three levels.

## 4. Experiment and Analysis

In this section, we define the normalization of input and output variables, selection of data sources and network parameters, and determination of BP network verification model in depth.

### 4.1. Normalization of Input and Output Variables

When processing data with a neural network model, it is generally necessary to preprocess the data, and the most commonly used processing method is data normalization. The data normalization processing method refers to converting all input and output data to between 0 and 1 on the basis of ensuring that the characteristics of the data information remain unchanged. The reason for normalizing the data is that since the neural network often deals with nonlinear functions, it can be seen in chapter 3, principles of network algorithms, that the nonlinear process is realized by the activation function of the network. The most commonly used activation function is the sigmoid function whose value range is [0, 1]. In the case of not normalizing the data, there may be a certain order of magnitude difference in the data, and the difference may be large. At this time, the data with a small value will produce small errors, while the data with a large number will produce a relatively large error. Also mentioned above, the training process of the neural network is based on the total error to adjust the weight of the neural network, which will cause the component with small error to account for a larger proportion of the total error than the component with large error in the total error. This is not conducive to the optimization of the network within a certain number of iterations. Normalizing the data can greatly reduce the impact of this problem on the model accuracy, which has been proved by the research of many scholars. Commonly used data normalization methods are mainly divided into maximum and minimum methods. Its normalization formula is as follows:

(14) $$\begin{array}{c} I=\frac{I-I_{\min}}{I_{\max}-I_{\min}}, \end{array}$$

where *I*_max_ and *I*_min_ are the maximum and minimum values in the data sequence to be processed, respectively.

### 4.2. Selection of Data Sources and Network Parameters

According to the evaluation indicators constructed in chapter 3, this paper designs a related questionnaire and then uses the big data technology to obtain the data set required for the experiment, including 280 sets of data, of which 240 sets are used as training sets and 40 sets are used as test sets. The number of nodes in the hidden layer is another important parameter of the hidden layer, but the precise determination of the number of nodes is still a key problem to be solved so far. Similar to the number of hidden layers, the selection of points also has the same problem. Too few nodes will affect the learning ability of the network and cannot achieve the expected accuracy. Too many nodes will not only increase the training time but also may cause the network to fall into a local optimal solution. According to the successful cases studied by relevant scholars, the selection of the number of nodes is usually given by the following empirical formula:

(15) $$\begin{array}{c} H=\sqrt{m+n}+a, \end{array}$$

where *H* is the number of nodes in the hidden layer, *m* is the number of neurons in the input layer, *n* is the number of neurons in the output layer, and *a* is a constant between 0 and 10.

The number of hidden layer nodes is estimated to be in the range of [4–14] using the algorithm above. As a result, the experiment is conducted using the trial and error approach, with the number of nodes chosen as 4, 6, 8, 10, 12, and 14 for the experiment. The results obtained are shown in Figures 2–4. Finally, according to the experimental results, the most suitable number of nodes is selected as 10.

### 4.3. Determination of BP Network Verification Model

The number of hidden layer nodes of the network model is 10, the number of input indicators is 10, and the test set is used for experiments. At this time, the actual output and expected output of the model are shown in Table 2. The network error is low, and the average prediction accuracy of the model is high. At this time, the network performance of the model is better, and the functional relationship between input and output can be approximated with high precision.

## 5. Conclusion

As a legal phenomenon, traditional customary law plays a role similar to that of national law in the formation of order and the settlement of disputes. It is closely related to national law in various fields and has an important influence on contemporary legal practice. However, to some extent, the legal circle of our country only regards customary law as a historical phenomenon or a manifestation of backward legal system, which is a misunderstanding in the study of customary law. If customary law is a social order that emerges spontaneously, it is acknowledged by academics as having had a significant historical impact, as evidenced by a great number of historical and sociological research findings. The worth of conventional customary law is assessed using a neural network in this paper. The work done is as follows:

1. This paper clarifies the concept of customary law and the difference between it and related concepts, and introduces domestic and foreign research on traditional customary law and dynamic legal practice. The status and effect of customary law in current legal practice is proposed by the interaction link between customary law and national law
2. The related technologies of neural network are introduced and a traditional customary value evaluation system that can be used for experiments is constructed
3. Experiment with the designed data set to see if the BP model is feasible. The experimental results suggest that the model proposed in this study has a low error rate and performs well while evaluating traditional common law values

## Figures and Tables

**Figure 1:** Schematic diagram of BP neural network structure.

**Figure 2:** Training effect when *N* = 4 and *N* = 6.

**Figure 3:** Training effect when *N* = 8 and *N* = 10.

**Figure 4:** Training effect when *N* = 12 and *N* = 14.

**Table 1:** Traditional and customary law value assessment system.

Number	Index	Label
1	Maintain the creative spirit of a nation	X1
2	Prevent social disputes in rural areas	X2
3	Liveness of content	X3
4	Informality of procedure	X4
5	Territoriality of jurisdiction	X5
6	Operational internal control	X6
7	Maintained constancy	X7
8	Politically significant	X8
9	Contribute to the construction of sound laws	X9
10	Contribute to regional economic benefits	X10

**Table 2:** The comparison between the expected output and the actual output.

Number	1	2	3	4	5	6	7	8
Actual output	0.815	0.728	0.691	0.885	0.762	0.785	0.693	0.919
Expected output	0.808	0.712	0.712	0.840	0.755	0.791	0.674	0.902
Error	0.007	0.016	0.021	0.045	0.007	0.006	0.019	0.017

## Data Availability

The datasets used during the current study are available from the corresponding author on reasonable request.
